# The Role of Muscle in Insect Energy Homeostasis

**DOI:** 10.3389/fphys.2020.580687

**Published:** 2020-10-22

**Authors:** Heidi Bretscher, Michael B. O’Connor

**Affiliations:** Department of Genetics, Cell Biology and Development, University of Minnesota, Minneapolis, MN, United States

**Keywords:** insect, muscle, energy, homeostasis, glycogen, lipids, signaling

## Abstract

Maintaining energy homeostasis is critical for ensuring proper growth and maximizing survival potential of all organisms. Here we review the role of somatic muscle in regulating energy homeostasis in insects. The muscle is not only a large consumer of energy, it also plays a crucial role in regulating metabolic signaling pathways and energy stores of the organism. We examine the metabolic pathways required to supply the muscle with energy, as well as muscle-derived signals that regulate metabolic energy homeostasis.

## Introduction

Regulating energy utilization and storage is essential for proper development and environmental adaptation. A constant supply of diet derived energy is required to sustain healthy cellular functions. Organisms must also maintain energy stores for times when nutrients are scarce as well as to fuel periods of high-energy expenditure, such as movement or flight. While energy stores are vital to survival, they must be tightly regulated as excessive or insufficient energy reserves are deleterious to survival and organismal health. In fact, excess energy stores are associated with many human metabolic diseases, obesity, cardiovascular disease and diabetes making the study of energy homeostasis of great interest to human health.

Energy homeostasis requires coordination of multiple organ systems, which communicate through many well-characterized cell signaling pathways. For example, in mammals insulin and glucagon are two well-conserved pathways that are crucial to energy homeostasis. Under nutrient rich conditions the hormone insulin is secreted from pancreatic beta cells. Insulin signals through the insulin receptor resulting in activation of two important pathways: the Mitogen-activated Protein Kinase (MAP-Kinase) and the Phosphatidylinositol-3-Kinase (PI3K). Activation of the MAP-kinase pathway results in cell mass increase through transcriptional upregulation of cell growth genes. The PI3K pathway has several functions, the most important being to signal glucose uptake as well as energy storage. Energy is stored in two main forms: glycogen and lipids. Glycogen is composed of long branched chains of glucose and is stored primarily in the liver and skeletal muscle. Lipids are synthesized from nutrient-derived carbons and stored primarily in adipose tissue as chains of varying lengths connected by a glycerol backbone. These energy stores become important under limited nutrient conditions or periods of increased energy demand. During these periods, insulin secretion decreases and secretion of a second hormone, glucagon, from pancreatic alpha cells increases. Glucagon signals through a G protein coupled receptor (GPCR) leading to mobilization of stored glycogen and lipids in a form that can fuel ongoing energy needs. These two signaling pathways are key to maintaining energy homeostasis of the whole organism and are conserved from mammals to insects.

In recent years *Drosophila melanogaster* has emerged as a model for studying metabolic homeostasis. Like many organisms, Drosophila relies on insulin and glucagon signaling to maintain energy balance. In this species, insulin like peptides (dILPs) are secreted from several sources, most importantly the Insulin Producing Cells (IPCs) in the brain. Upon secretion, dILPs bind the insulin receptor (InR) activating the MAP-kinase and PI3K pathways with similar downstream targets to mammals (Nässel et al., 2013; Mattila and Hietakangas, 2017). Conversely, in times of limited nutrients adipokinetic hormone (Akh), a functional glucagon homolog, signals through its corresponding GPCR (AkhR) and leads to energy mobilization (Grönke et al., 2007; Bharucha et al., 2008; Gáliková et al., 2015). Like mammals, *Drosophila* store energy in the form of lipids and glycogen. Lipids are found primarily in the fat body, which is analogous to mammalian adipose tissue and liver, while glycogen is found in skeletal muscles as well as fat body and the central nervous system. Again, analogous to mammals, these energy reserves are essential not only for times when nutrients are scarce, but also for times of increased energy demand such as movement or flight. The high degree of genetic conservation between mammalian and *Drosophila* metabolic pathways, the extensive genetic tool kit available in *Drosophila* and short generation time, makes *Drosophila* an ideal model to study regulators of metabolic and energy homeostasis. In addition, *D. melanogaster* are generalists and can thus be raised on a flexible diet enabling study of gene-diet interactions. *Drosophila* have emerged as a model for studying genetic and dietary forms of Type 2 Diabetes (Musselman et al., 2011) as well as glycogen storage diseases (Zirin et al., 2013).

In most triploblastic organisms, muscle is the largest organ by weight and can account for up to 50% of the adult mass. The major function of muscle is to enable movement to find food, escape predation, and initiate courtship behavior. As a consequence, it is the largest consumer of energy. Insect flight is a one of the most metabolically demanding processes in the animal kingdom. During flight, oxygen consumption increases one-hundred fold (Eanes et al., 2006). Thus, it is not surprising that somatic muscle plays an important role in regulating energy stores as well. Here we review the role of *Drosophila* skeletal muscle as an energy consumer and as an organ that regulates energy storage, and modulates insulin signaling.

## The Skeletal Muscle Is a Large Consumer of Energy

Insect flight is a truly incredible process and has been a source of fascination and study for more than seven decades. Adult flight is powered by direct flight muscles (DFMs) and indirect flight muscle (IFMs), which are found in the thorax. IFMs are capable of producing a mechanical force of just under 80 W kg^–1^ during flight (Lehmann and Dickinson, 1997). A separate set of muscles, known as jump muscles, are located in the legs and give the animal the ability to walk and jump. Adult body wall muscle is similar in structure to vertebrate counterparts, being tubular in shape. However, unlike the adult, larval body wall muscles are largely two-dimensional one cell thick thin sheets. Most larval muscles are histolyzed during metamorphosis and replaced by adult muscles that are derived from adult muscle founder cells (Gunage et al., 2017). A more detailed description of *Drosophila* muscle types and function has been thoroughly reviewed previously (Bernstein et al., 1993). Despite being among the most metabolically demanding processes in the animal kingdom, 1 week old *Drosophila* can sustain flight for an average of 278 min (Wigglesworth, 1949). Upon flight initiation, glucose is consumed in approximately 2 min (Sacktor and Worbber-Shavit, 1966). While this is associated with a temporary dip in glucose levels, they soon return to a steady state, which is maintained during flight (Sacktor and Worbber-Shavit, 1966). The main source of glucose used to power flight is glycogen, and glycogen stores are readily mobilized during flight and almost depleted in flies flown to exhaustion (Wigglesworth, 1949). Upon exhaustion, supplying flies with a glucose solution allows a return to flight within 30–45 s, whereas other carbohydrates, such as lactose and xylose, require longer time intervals to take effect, suggesting that glucose is the main fuel source for the muscle (Wigglesworth, 1949). In addition to glucose, muscles also readily utilize trehalose, an insect specific carbohydrate that is synthesized in the fat body (Sacktor and Worbber-Shavit, 1966). Trehalose is composed of two glucose molecules linked by a glucoside linkage and can be transported into skeletal muscle and cleaved into two glucose molecules (Shukla et al., 2015). Trehalose is also a vital fuel source during eclosion, as flies unable to synthesize trehalose die during the eclosion process (Matsuda et al., 2015). Thus, glucose, and trehalose are vital sources of energy for muscles. Despite the fact that the original research on glucose and glycogen consumption during flight was conducted over 70 years ago, (Wigglesworth, 1949) the signals required for glycogen mobilization upon flight initiation remain ill-defined. Furthermore, the role of lipids in powering flight in *Drosophila* is an area that requires further study.

In several insect species, including cockroaches and migratory locusts (*Locusta migratoria*), Akh is released upon flight initiation (Gäde et al., 1997). This results in mobilization of fat body glycogen stores, leading to increased hemolymph trehalose levels needed to supply increased energy demands by muscle. While some insects, including flies and cockroaches, rely primarily on carbohydrates to fuel flight, stored lipids are an important fuel source for locusts (Gäde et al., 1997). In locusts, Akh release results in fat body lipid mobilization and increases the lipid carrying capacity of the hemolymph by activating lipoproteins (Gäde et al., 1997; Van Der Horst, 2003). Fatty acids derived from hemolymph lipids can be oxidized by muscles of locusts and used for energy (Van Der Horst, 2003). Interestingly, in *Drosophila*, Akh appears to be dispensable for flight performance and climbing ability (Gáliková et al., 2015). In fact, the Akh receptor, AkhR, is expressed mainly in fat body and gustatory neurons and not muscle (Yoshida et al., 2016). Additionally, Akh is dispensable for the mobilization of glycogen and lipids during development. However, Akh does play a role in carbohydrate homeostasis as both larvae (Lee and Park, 2004) and adult (Gáliková et al., 2015) Akh mutants have lower levels of hemolymph trehalose (Lee and Park, 2004; Gáliková et al., 2015). In light of the role of Akh in mobilizing energy for flight in other insects, as well as its role in maintaining trehalose levels in *Drosophila*, it is interesting that Akh does not appear to affect *Drosophila* flight performance.

In *Drosophila* and other related insects, muscles rely primarily on aerobic glycolysis to convert glucose and other carbohydrates into energy. Glycolysis occurs in the cytoplasm of muscle cells and consists of a series of enzymatic reactions that convert glucose into two molecules of pyruvate and two ATP molecules per molecule of glucose (Figure 1). The majority of energy is derived from the TCA/Krebs Cycle, which occurs in the matrix of the mitochondria (Sacktor and Worbber-Shavit, 1966). Pyruvate enters the mitochondria and is converted to Acetyl-CoA (Figure 1). Acetyl-CoA is oxidized in a series of chemical reactions generating CO_2_, ATP and a pool of NADH and FADH_2_ (Figure 1). NADH and FADH_2_ are then oxidized in a process known as oxidative phosphorylation. The majority of energy from this process is stored as an electrochemical gradient and used to power ATP synthase (Figure 1). ATP is then supplied to the myosin ATPase enabling muscle contraction. Disrupting this process in muscle can affect the ability of muscle to function optimally (Wojtas et al., 1997).

**FIGURE 1:** The muscle stores and consumes energy. The muscle stores energy in the form of glycogen. Glycogen consists of long chains of glucose and is synthesized by GlyS. Glycogen can be broken down by GlyP or via autophagy to provide the muscle with energy in times of need. When energy is needed glucose enters glycolysis, a series of enzymatic reactions which occur in the cytoplasm to form two molecules of pyruvate and ATP. The majority of pyruvate enters the inner matrix of the mitochondria where it is converted to Acetyl-CoA and oxidized in the TCA cycle producing NADH and FADH_2_. NADH and FADH_2_ power oxidative phosphorylation which creates an electrochemical gradient used to power ATP synthase producing ATP.

Glycolysis is necessary for maximal wing beat frequency as inhibition of glycolysis reduces wing beat rate (Eanes et al., 2006). Most glycolytic enzymes, with the exception of hexokinase and phosphoglycerate mutase (PGM) (Figure 1) are present in excess, as reductions in enzymatic expression levels do not alter wing beat frequency (Eanes et al., 2006). Glycolytic enzymes in muscle are located in distinct patterns enabling resulting ATP to be supplied to the myosin ATPase. Incorrect localization of enzymes results in decreased flight ability (Wojtas et al., 1997) highlighting the importance of aerobic glycolysis in powering flight.

Aerobic glycolysis is not limited to adult flies, but is also required for proper larval development. During larval stages, animals increase in size roughly two hundred fold in a matter of days, and body wall muscle must increase in size rapidly in order to power larval locomotion. Again aerobic glycolysis is required to sustain the energetically expensive process of growth. Larvae mutant for proteins important for stabilizing the glycolytic enzymes aldolase and PGM show decreased glycolytic flux resulting in decreased amino acid pools and decreased ATP levels (Bawa et al., 2020). This results in small degenerated muscles, thus underscoring the importance of this process in fueling proper development and growth (Bawa et al., 2020). Similarly, lack of the glycolytic enzyme phosphoglycerate mutase 2 (pgam2) results in abnormally thin muscles (Tixier et al., 2013).

Unlike mammals, flies do not typically rely on anaerobic respiration, a process by which pyruvate is converted to lactate in the cytoplasm (Feala et al., 2007; Figure 1). Interestingly, this makes flies remarkably resistant to hypoxic and even anoxic conditions. While humans can survive for only minutes in anoxia, flies can survive for up to 4 h (Feala et al., 2007). Increased survival time for flies is due to lack of lactate build up. Rather than converting pyruvate to lactate, flies covert pyruvate to alanine and acetate, which are less acidic and more energetically favorable than lactate (Feala et al., 2007). In addition, levels of proline and glutamine decrease indicating that amino acids are being broken down and entering the Krebs cycle (Sacktor and Worbber-Shavit, 1966; Feala et al., 2007). These findings suggest that rather than relying on cytoplasmic lactate production, flies utilize the mitochondria and the Krebs cycle to power muscle movement in times of hypoxic stress.

Given the importance of the Krebs cycle in energy production in the muscle, it is no surprise that mitochondria are also central to maintaining energy homeostasis. In larvae, disrupting mitochondrial activity results in decreased oxygen consumption, decreased ATP production, and smaller muscles (Song et al., 2017). During the first 7 days of adulthood, muscle mitochondrial area increases, which is correlated with maximal flight performance (Sohal, 1975). Mitochondria are very dynamic structures and undergo fission and fusion, which are necessary for both quality control and energy production. During the first 7 days of adulthood, mitochondria increase size by growth as well as fusion (Wigglesworth, 1949). As flies age, total area occupied by mitochondria remains steady, but fission occurs resulting in smaller mitochondria. Decreased mitochondrial size is enhanced in dewinged flies (Sohal, 1975). This observation suggests that exercise may be required to maintain mitochondrial structure in older adults, however, the relationship between exercise and mitochondrial function remains a notable area for further study.

Mitochondrial fission and fusion require expression of nuclear encoded genes, which are regulated by the nuclear encoded transcription factor Ewg (mammalian NRF1 homolog). Loss of Ewg results in decreased expression of Optic atrophy 1 (Opa1), which is required for inner membrane fusion (Rai et al., 2014), resulting in smaller rounded mitochondria that co-localize with the lysosome suggesting that they are undergoing mitophagy. The smaller mitochondrial structure leads to abnormal muscle development during pupation. As adults, animals mutant for Ewg, and therefore expressing lower levels of Opa1, show a decreased number of IFMs and disorganized DLMs (Rai et al., 2014). Taken together these findings demonstrate that muscle mitochondrial fission and fusion is required for proper pupal development and adult muscle function.

The inner mitochondrial membrane contains many cristae, or folds, that maximize surface area, allowing for efficient electron chain transfer and ATP production. Cristae structure is maintained by the mitochondrial contact site and cristate organizing system (MICOS) (Yoon et al., 2019). MICOS is activated by the ATPase YME1 like ATPase (YME1L), and YME1L in turn is activated by the serine/threonine kinase aarF domain containing kinase (dADCK1). Thus, loss of dADCK1 results in lack of YME1L 1 and MICOS activation. dADCK1 mutant animals are delayed in development and are small in size demonstrating the importance of mitochondria in fueling the growth process (Yoon et al., 2019). While dADCK1 mutants are lethal, depleting dADCK1 specifically in the muscle results in viable adults with abnormal mitochondrial structure, decreased mitochondrial surface area and decreased mitochondrial membrane potential resulting in decreased ATP pools. Lack of sufficient ATP leads to decreased wing movement and abnormal wing posture, demonstrating the importance of mitochondrial cristae in providing the muscles with energy to power wing movement and flight (Yoon et al., 2019).

Mitochondria also play an important role in maintaining energy homeostasis when responding to different nutrient sources. Specifically, mitochondria are flexible as to the substrates that enter the electron transfer chain based on availability. However, metabolic overload can overwhelm mitochondria and reduce this flexibility (Cormier et al., 2019). For example, animals fed on a high fat diet (HFD), become reliant on a single mitochondrial membrane complex for entry into the electron transfer chain (Cormier et al., 2019) and are limited in the types of substrates that can be oxidized. Metabolic overload and lack of mitochondrial flexibility ultimately brings about decreased ATP in the thoracic muscle as well as decreased climbing ability and a decreased lifespan. In addition to lower ATP, muscles were found to have decreased levels of stored energy, likely contributing to decreased muscle performance (Cormier et al., 2019). This demonstrates that muscles are not only active consumers of energy but also must store some of their own energy to mobilize in times of need. Given the ease of diet manipulation, it is surprising that more studies have not investigated the relationship between specific diet components and locomotor behavior in larvae or adults.

## Skeletal Muscles as a Source of Stored Energy

Given the intense energy demands of insect muscle, it is no surprise that muscles are also an important source of stored energy in the form of glycogen (Yamada et al., 2018, 2019; Figure 1). Glycogen consists of long branched chains of glucose synthesized by the enzyme glycogen synthase (GlyS) (Figure 1). Synthesis of glycogen from dietary glucose in the fat body requires insulin signaling (Yamada et al., 2018) and animals lacking dILP1 (Liao et al., 2020), dILP2, or dILP5 have lower whole body glycogen levels (Post et al., 2018). However, the relationship between insulin signaling and glycogen storage in the muscle has not been studied. Insulin resistance resulting from a high sugar diet leads to lower glycogen levels despite elevated hemolymph sugars in both larvae (Musselman et al., 2011) and adults (Morris et al., 2012), but again whether this difference is limited to just fat body glycogen levels or also affects muscle glycogen levels is unknown.

Glycogen is broken down by glycogen phosphatase (GlyP) (Figure 1) to liberate free glucose molecules used to power movement and flight. GlyP is negatively regulated by insulin signaling, specifically by dILP2 (Post et al., 2018). In many insects, Akh is important for activating GlyP upon flight initiation (van Marrewijk et al., 1986; Van Der Horst, 2003). During times of high demand, GlyP works at near saturation as small alterations in GlyP levels results in decreased wing beat frequency (Eanes et al., 2006). However, the signal that activates GlyP in *Drosophila* upon flight initiation is unlikely to be Akh (Grönke et al., 2007; Bharucha et al., 2008; Gáliková et al., 2015) and its identity is an important goal that remains to be determined.

Glycogen is an important fuel source throughout development. Most animals lacking GlyS, and thus unable to synthesize glycogen, die as larvae; however, a few make it to adulthood. Larval survival of GlyS mutants can be increased by a high yeast, high glucose diet, but many of these animals die during metamorphosis (Yamada et al., 2019). In larvae, glycogen is primarily stored in body wall muscles, but is also found in the fat body and CNS. Lack of GlyS in the muscles results in a significant decrease in survival rate, similar to that of a GlyS mutant, while loss of GlyS in the fat body does not affect survival (Yamada et al., 2018). While not required for survival, fat body stores of glycogen can fuel the animal through brief periods of starvation and has thus been termed a “metabolic safeguard” (Yamada et al., 2018). In the fat body, glycogen can be either converted directly to glucose, or used to synthesize trehalose. Trehalose is secreted from the fat body, and can be used by other tissues, such as the muscle. Once in the muscle, trehalase breaks down trehalose into glucose which can be used as an energy source (Yoshida et al., 2016). In the fat body glycogen breakdown occurs mostly by GlyP (Zirin et al., 2013). However, starvation induced glycogen breakdown in the muscle can occur either through GlyP or autophagy. Inhibiting either process alone does not prevent starvation induced glycogen breakdown, however, inhibiting both simultaneously prevents starvation induced glycogen breakdown in the muscle (Zirin et al., 2013). In the fat body, starvation induced autophagy requires inhibition of the Tor kinase pathway. While the link between Tor activity and insulin signaling in muscle has not been fully explored, it is tempting to speculate that it is reduced insulin signaling upon starvation that inhibits Tor activity. Inhibition of both GlyP and autophagy also results in reduced crawling speeds following periods of starvation underscoring the importance of glycogen as a fuel source for the muscle in sustaining movement (Zirin et al., 2013). It would be interesting to know whether Tor activity modulates the activity of GlyP, or just starvation induced autophagy.

In addition to being important for larval survival and larval locomotion, glycogen is a key source of stored energy in adult muscle. In adults, glycogen is also stored in the fat body, halteres, proventriculus and midgut (Wigglesworth, 1949). Glycogen stores peak at 1 week in age, which is correlated with maximal flight performance (Wigglesworth, 1949). Decreased flight performance and climbing speeds are seen in animals lacking GlyS or GlyP highlighting the importance of glycogen in physical fitness (Yamada et al., 2019). However, these animals can still climb and fly indicating that some level of compensation for lack of glycogen stores must be occurring. Due to changes in levels of glucogenic amino acids in GlyS and GlyP mutants, it has been speculated that these mutants have altered amino acid metabolism (Yamada et al., 2019). Loss of both GlyS and GlyP also results in decreased trehalose levels since glycogen is often used to synthesize trehalose (Yamada et al., 2019). Trehalose is an important fuel source for muscles, and animals hypomorphic for trehalose-6-phosphate synthase (Tps1), which is required for trehalose synthesis, also demonstrate reduced flight and climbing performance (Matsuda et al., 2015).

While enzymes involved directly in carbohydrate metabolism have clear roles in maintaining carbohydrate homeostasis, homeostasis is also affected by other factors. In order to synthesize glycogen, animals must digest dietary carbohydrates to form glucose. Digestion begins in the midgut where amylases are secreted into the gut lumen. Expression of these amylases is tightly regulated and is controlled in part by the nuclear receptor DHR38 (Ruaud et al., 2011). Animals lacking DHR38 have reduced expression levels of two digestive amylases as well as phosphoglycomutase that result in reduced glycogen stores in the muscle highlighting the importance of these enzymes in maintaining glycogen homeostasis (Ruaud et al., 2011). On the flip side, amylases are inhibited by high dietary sugar via the transcription factor Sugarbabe (Mattila et al., 2015). Metabolic overload, such as a high sugar diet, leads to reduced glycogen stores (Musselman et al., 2011; Morris et al., 2012), further emphasizing the importance of nutrition in maintaining energy homeostasis. The transcription factor missing oocyte (Mio) (ChREBP homolog) also regulates the expression of genes required for utilization of diet derived fuel sources. In the muscle, Mio is important for glycogen utilization since animals lacking Mio in the muscle have increased glycogen levels (Polak et al., 2015). Loss of Mio in the muscle also leads to small and disorganized myofibrils with irregular spaces filled with glycogen granules. As a result, increased glycogen granules and abnormal muscle structure contribute to decreased flight performance as observed in animals lacking Mio expression in the muscle (Polak et al., 2015). Given the importance of glycogen stores for muscle function, it seems likely that additional genes beside dILP2 (Post et al., 2018), DHR38 (Ruaud et al., 2011), and Mio (Polak et al., 2015) are required to modulate levels of muscle glycogen stores and screens to identify them should prove fruitful.

## The Role of Muscle in Maintaining Lipid Homeostasis

Under normal conditions, lipids/triacylglycerol (TAG) are not found in muscle but are stored mainly in fat body and oenocytes (Heier and Kühnlein, 2018). Ectopic fat accumulation in muscle is associated with insulin resistance, muscle weakness and structural abnormalities and is seen with dietary or genetically induced obesity (Villanueva et al., 2019). Obese animals also have disorganized myofibrils and mitochondrial damage leading to an accelerated age related decrease in climbing rate. Interestingly, accumulation of lipid droplets in the muscle of obese flies can be rescued by time restricted feeding (Villanueva et al., 2019). In addition to obesity, age is also associated with lipid droplet accumulation in muscles, especially jump muscles (Yan et al., 2017). Increased lipid droplets in aged flies are a result of an increase in Perilipin 2 (PLIN2), which has been shown to protect lipid droplets. In young flies, PLIN2 levels are modulated through the activity of histone deacetylase 6 (HDAC6) and the chaperone Heat shock 70 kDA protein cognate 4 (Hsc4) that mediate ubiquitin-proteasomal and lysosomal degradation of native and/or misfolded proteins. HDAC6 expression decreases with age, thereby effecting an increase in PLIN2 and subsequent lipid droplet accumulation in muscle (Yan et al., 2017). Increased insulin signaling in the muscle also results in the presence of TAGs in the muscle of adult flies, while decreasing TAGs elsewhere (Zhao and Karpac, 2017). Insulin signaling typically represses the transcription factor forkhead box subgroup O (FoxO). Loss of FoxO in the thoracic skeletal muscle results in the appearance of lipids in the muscle and upregulation of the cytokine unpaired 2 (upd2). This in turn leads to increased Akh secretion, mobilization of lipid, and decreased TAGs in the fat body and gut, despite having ectopic lipid accumulation in the muscle (Zhao and Karpac, 2017). This demonstrates that while lipids are usually absent in the muscle, the muscle can be an important regulator of lipid levels. It is interesting that both insulin resistance and increased insulin signaling in muscle result in ectopic lipid accumulation, suggesting that a very precise level of insulin signaling is needed in muscle to suppress muscle TAG accumulation.

While muscles do not typically store lipids, myokines serve as important regulators of organismal lipid stores. Lipid stores in the fat body of adults are regulated in response to muscle derived Wingless (Wg), the expression of which requires muscle Med13, part of the complex that regulates interactions between RNA Pol II and transcription factors (Lee et al., 2014). Lack of either Med13 or Wg in muscle produces increased TAGs in fat body, increased lipid droplet size and starvation resistance. Interestingly, loss of Med13 or Wg in either the skeletal muscle or cardiac muscle is sufficient to increase TAG levels (Figure 2). A second myokine that has been shown to suppress obesity is the PDGF/VEGF ligand Pvf1. However, unlike Wg that signals to the fat body, Pvf1 signals to the oenocytes, a specialized hepatocyte like cell. Oenocytes express the Pvf1 receptor PvR, and activation of PvR in oenocytes results in activation of mTOR which in turn leads to increased PI3K and Akt. This Pvf1-mTOR-Akt signaling cascade from muscle to oenocytes slows the rate of lipid synthesis without affecting the rate of lipid mobilization (Ghosh et al., 2020; Figure 2). The rate of lipid synthesis is very rapid in young flies, and Pvf1 expression levels are found to be very low at the time of eclosion. Overexpression of Pvf1 in young flies results in inhibition of developmentally programmed TAG synthesis (Ghosh et al., 2020). Future studies will be needed to elucidate the signal between oenocytes and fat body in response to muscle derived Pvf1.

**FIGURE 2:** The muscle regulates TAG storage and insulin signaling. Signaling pathways from and to the muscles affect metabolic homeostasis. Actβ and Dawdle are Activin-like members of the TGFβ superfamily of signaling factors. JAK/STAT factors are signal transduction components that act downstream of insect Unpaired ligands. TIF-IA is a transcription factor that connects RNA polymerase I with the UBF/SL-1 complex to initiate the transcription of pre-ribosomal RNA. Med13 is a member of the Mediator Complex a transcriptional coactivator complex. Pvf1 is an insect PDGF/VDGF homolog. IMPL2 is an insect insulin binding protein. Nep4A is a muscle localized Neprilysin that likely is responsible for cleavage of the several neuroendocrine peptides including DH31, Allatostatin A, tachykinin, and Neuropeptide F are derived from the gut that regulate insulin secretion from the brain.

While loss of Wg signaling or Pvf1 in muscle increases TAG levels, loss of cytokine activated Janus Kinase/signal transducer and activator of transcription (JAK/Stat) signaling in muscle decreases TAGs (Kierdorf et al., 2020; Figure 2). This dynamic is mediated through increased p-AKT levels and thereby increased insulin signaling. In addition to decreasing TAGs, loss of JAK/Stat and the consequent increased insulin signaling leads to TAG presence in the muscle and decreased total glucose and glycogen levels in the organism, likely resulting from an increased metabolic rate (Kierdorf et al., 2020). This result is similar to what was seen with loss of FoxO, a negative regulator of insulin signaling, which also results in ectopic lipid accumulation in muscle (Zhao and Karpac, 2017). Interestingly, this report also found an upregulation of the JAK/Stat ligand Upd2 in the muscle of animals with increased insulin signaling. It would be interesting to know whether Upd2 may be able to signal back to the muscle to reduce insulin signaling. Finally, in larvae, increased expression of the Transforming growth factor-beta (TGF-β) ligand Activin-β in the muscle generates increased free fatty acids, organismal TAGs and TAG storage in the fat body (Figure 2). Activin-β signals through a heterodimeric receptor composed of Baboon and Punt, which are found in the fat body, increasing TAG storage (Song et al., 2017).

Despite the fact that TAGs are not stored in muscle, the muscle is still important in regulating TAG homeostasis as can be seen under conditions of dietary restriction. Dietary restriction has been shown to increase lifespan in many models, including *Drosophila*. In *Drosophila* dietary restriction is not associated with a decrease in total TAG levels, but conversely an increase in both total body TAG stores and lipid droplet size as well as the rate of both lipogenesis and lipolysis. The molecular mechanism by which lipolysis is increased is not known. It would be interesting to see whether dietary restriction changes the length or saturation level of stored TAGs, as this has been shown in other systems to alter the lipolysis rates (Benito-Gallo et al., 2015). In addition to increased TAG turnover, animals fed a restricted diet also demonstrate increased physical activity and improved muscle function (Katewa et al., 2012). These phenotypes are dependent on the enzyme Acetyl-CoA carboxylase (ACC). Interestingly, ACC in the fat body, the tissue where the majority of TAGs are stored, is not required to increase life span, but instead ACC in the muscle, a tissue that does not typically store TAGs is required for increased lifespan resulting from dietary restriction (Katewa et al., 2012). Why ACC expression would be required in the muscle and not the fat body remains to be determined. The muscle is clearly key to mediating the effects of dietary restriction as genome wide loss of ACC results in decreased expression of muscle structure and function genes. Furthermore, inhibiting physical activity of flies by ablating or clipping wings significantly reduced the effects of dietary restriction on increased lifespan (Katewa et al., 2012). These results demonstrate that the muscle is a key tissue for responding to dietary restriction, but do not address the question of what specific role ACC might play in muscle. Since dietary restrictions results in increased TAG turnover (Katewa et al., 2012), it would be interesting to see if TAGs transport to muscles is required for the increased lipolysis. Furthermore, this study looked only at TAG levels in response to dietary restriction and did not consider glycogen, another important form of stored energy. It would be interesting to see whether glycogen stores in muscle and or fat body are altered by dietary restriction.

## The Skeletal Muscle Modulates Insulin Signaling

Proper growth of muscles is dependent on insulin signaling. Lack of insulin signaling in muscle results in smaller muscle size and decreased nuclear ploidy (Demontis and Perrimon, 2009). Decreased size is due to lack of insulin dependent inhibition of the transcription factor FoxO. Increased FoxO activity results in inhibition of dMyc expression, which is required for muscles to reach normal size and nuclear ploidy (Demontis and Perrimon, 2009). FoxO dependent regulation of myc is also important in response to low nutrient conditions. In the muscle, inhibition of myc by FoxO results in decreased protein translation, presumably to conserve energy (Teleman et al., 2008). Insulin signaling in larval muscles is regulated by other signaling pathways including the TFG-β/Activin signaling pathway ligand Activin-β. Activin-β positively regulates insulin signaling and is required for proper muscle geometry and sarcomere protein level (Kim and O’Connor, 2020). While these studies show the importance of insulin signaling in proper muscle size and structure, whether insulin signaling in the muscle alters levels of stored glycogen locally or globally is unknown. This is surprising given the importance of insulin signaling in maintaining carbohydrate homeostasis.

The JAK/Stat and insulin signaling pathway cooperate in larval muscle to mount an immune response. Fighting infections is an energetically expensive process. Following parasitic wasp infection hemocyte derived Upd2 and Upd3 activate JAK/Stat signaling in muscle, which in turn increases insulin signaling (Yang and Hultmark, 2017). This process is fueled by glycogen stored in muscle. Thus, animals lacking sufficient muscle glycogen stores are more susceptible to infection (Yang and Hultmark, 2017). This is one of the only reports that clearly links muscle glycogen stores to a distinct function in larvae. Another report found that glycogen muscle stores were needed for optimal locomotor function under starvation conditions (Zirin et al., 2013). Interestingly, in adults, JAK/Stat signaling is required to prevent high levels of insulin signaling. JAK/Stat ligands Upd1, 2, 3 are supplied by plasmocytes and activate JAK/Stat signaling in muscle. Suppression of JAK/Stat signaling in adult muscle results in increased insulin signaling in muscle, which shortens life span and decreases climbing ability (Kierdorf et al., 2020). This may simply be a difference between larvae and adults, however, it may also suggest that both low and high levels of JAK/Stat signaling in the muscle can result in increased insulin signaling. It has been demonstrated that increased insulin signaling in muscle results in muscle upregulation of Upd2 (Zhao and Karpac, 2017). Whether Upd2 signals back to the muscle, and if so, does it positively or negatively regulate insulin signaling remains unclear.

As described above, insulin signaling to the muscle plays an important role in proper muscle growth and function. In addition to being a receiver of insulin signaling, the muscle modulates insulin signaling in the whole animal. During larval development, insulin signaling is coupled to the availability of nutrients via the TOR pathway, which is required for growth (Colombani et al., 2003). One way it does this is by increasing mRNA and protein levels of Transcription initiation factor-IA (TIF-IA), a transcription factor required for ribosomal synthesis (Ghosh et al., 2014). In addition to promoting muscle growth, TIF-IA also affects the level of insulin signaling. Loss of TIF-IA in the muscle results in decreased dILP3 and dILP5 mRNA levels, increased retention of dILP2 in the IPCs as well as increased expression of Imaginal morphogenesis protein-Late 2 (IMPL2), a negative regulator of insulin signaling (Figure 2). It remains unclear the mechanism by which TIF-IA in muscle affects transcription levels of dILPs or dILP release. It is worth mentioning that when TIF-IA expression was decreased in muscle using RNAi, resulting in the decrease in dILP transcription levels, the driver used (mef2 gal4) is not specific to the muscle, and also shows some expression in the CNS. Testing with additional specific-muscle only drivers seems warranted.

Overexpression of the transcription factor FoxO in muscle, which is negatively regulated by insulin signaling, results in repression of the TGF-β ligand Dawdle. Dawdle signals cell-autonomously to muscle through the TGF-β receptor Baboon, which activates the transcription factor Smox (Bai et al., 2013). Low insulin signaling therefore results in lower Smox activation and transcriptional upregulation of autophagic genes preserving muscle function and structure in older animals. In addition to affecting the muscle, increased Dawdle expression from the muscle gives rise to decreased dILP2 secretion and decreased insulin signaling (Figure 2). The combination of increased autophagic genes in the muscle and decreased insulin signaling in the whole animal results in an extended lifespan (Bai et al., 2013). However, a more recent study suggests that the role of muscle TGFβ signaling in regulating lifespan is more complicated since overexpression of either Dawdle or a second ligand Myoglianin in adult muscle appears to extend lifespan, in part, through enhanced production of the 26S proteasome (Langerak et al., 2018). Increased lifespan as a result of decreased insulin signaling can also be achieved through mild mitochondrial perturbation in larval muscle, which results in upregulation of IMPL2 in adults, which then binds to and inhibits dILPs (Owusu-Ansah et al., 2013; Figure 2).

Another way in which muscle is thought to modulate insulin signaling is via expression of the neprilysin Neprilysin4A (Nep4A), which can cleave and inactivate regulatory peptides. Overexpression of Nep4A in larval body wall muscle results in several phenotypes indicative of decreased insulin signaling including reduced body size, decreased food intake and increased glucose levels (Hallier et al., 2016). Indeed, overexpression of Nep4A in muscle reduces expression of dILPs 1,2,3, and 5. Given that Nep4 is found localized to the membrane of muscle cells suggests that Nep4A may cleave peptides that positively regulate insulin signaling. *In vitro* experiments found that Nep4A cleaves several peptides involved in dILP synthesis and/or feeding behavior including Allatostatin A, Neuropeptide F, DH31 and tachykinins 1,2,4, and 5 (Hallier et al., 2016). These peptides are produced in the CNS as well as by enteroendocrine cells in the midgut, leading the authors to speculate that Nep4A on muscle may cleave gut derived peptides as they travel through the hemolymph from the gut, thereby preventing them from reaching the IPCs (Figure 2). It is worth noting that Nep4A is also expressed in the CNS and is found localized to the membrane of IPCs. While neural or glial knockdown of Nep4A does not alter feeding behavior or body size, it is not clear if CNS expression of Nep4A may be important for cleavage of insulin promoting peptides, derived either from the gut or the CNS (Hallier et al., 2016).

## Concluding Remarks

While it has been appreciated for over half a century that insect muscle is a large consumer of energy (Wigglesworth, 1949; Sacktor and Worbber-Shavit, 1966), more recently the focus has shifted to the role of muscle in maintaining energy homeostasis (Katewa et al., 2012; Lee et al., 2014; Hallier et al., 2016; Song et al., 2017; Zhao and Karpac, 2017) and numerous avenues of investigation remain to be explored. One curious observation is that, while Akh signaling is required in several insects for maximal flight performance (Gäde et al., 1997; Van Der Horst, 2003), Akh seems to be dispensable for flight performance in *Drosophila* (Gáliková et al., 2015). What serves as the signal to the muscle that additional energy is needed upon flight initiation? It has been shown that muscle glycogen stores are necessary for maximal flight performance (Yamada et al., 2019). However, the signals that initiate breakdown of muscle glycogen stores during flight remain unknown. Furthermore, while several studies have focused on signals that regulate storage of fats in muscle and elsewhere, how glycogen storage is regulated in muscle and fat body remains largely unexplored.

Several reports have focused on how the muscle regulates insulin and Akh signaling at the organismal level (Hallier et al., 2016; Yan et al., 2017; Bawa et al., 2020). However, little is known about the effect of insulin and Akh signaling on energy storage in the muscle itself. While, it has been demonstrated that increased insulin signaling in the muscle can lead to ectopic lipid accumulation (Zhao and Karpac, 2017), the question of if and how insulin signaling regulates muscle glycogen stores remains to be determined.

One exciting new avenue that is being developed is the use of *Drosophila* as an exercise model. Worldwide, obesity rates are increasing and causing an increase in diseases associated with obesity, such as Type II diabetes, cardiovascular disease and kidney disease to name a few. One of the most prescribed treatments for obesity is increased physical exercise, yet the genetics behind the response to exercise remains largely unknown. Given that *Drosophila* has served as an excellent model for better understanding energy homeostasis, there has been a recent push to develop an exercise model for *Drosophila*. Thus far, a *Drosophila* Treadwheel (Lowman et al., 2018) has been developed as well as rotational exercise quantification system (Watanabe and Riddle, 2017). These new tools should enable exciting future work exploring how exercise affects muscle and the effects this has on organismal energy homeostasis.

## Author Contributions

HB conceived and wrote the manuscript. MO’C edited the manuscript and provided funding. All authors contributed to the article and approved the submitted version.

## Conflict of Interest

The authors declare that the research was conducted in the absence of any commercial or financial relationships that could be construed as a potential conflict of interest.
